# Prediction and Evaluation Method of e-Commerce Service Satisfaction Based on Intelligent Computing Method

**DOI:** 10.1155/2022/2730660

**Published:** 2022-08-30

**Authors:** Fang Tu, Bo Tu

**Affiliations:** ^1^Jiangxi Engineering Vocational College, Jiangxi Open University, Jiangxi 330046, China; ^2^School of Art East Jiao Tong University, East China Jiaotong University, Jiangxi 330013, China

## Abstract

Among the many service industries, e-commerce, which is based on the Internet and relies mainly on platforms and third-party transaction models, has developed rapidly. All localities have actively deployed their regional e-commerce development strategies to improve the core competitiveness of the regional economy. The rapid development of e-commerce provides a favorable development environment and construction environment for the spatial agglomeration of e-commerce service industry. We use the intelligent computing method to calculate the e-commerce service degree prediction experimental results that show that according to the curves of the three algorithms, we can also see that the curve values of the intelligent computing and fuzzy statistical algorithm models are very stable and the experimental results are also very stable. It shows that the performance of the intelligent computing algorithm is the most superior; the second-level indicators are the after-sales service of the merchant, the popularity of the merchant, and the attitude of the merchant's customer service; in the establishment of the logistic satisfaction evaluation index system, we found that the logistic satisfaction is the first-level indicator; the secondary indicators are the speed of logistics, the safety of logistics, the service attitude of logistics, and the price of logistics; after running on the test set, the model accuracy rate of the fuzzy statistical algorithm is 89.12%, and the accuracy rate can reach 89.56%. The accuracy rate of the intelligent algorithm can reach 92.46%, and the accuracy rate can reach 93.27%, which is the one with the highest index value among the three experimental models. Among the many service industries, e-commerce, which is based on the Internet and relies on platforms and third-party transaction models, is developing rapidly. All localities have actively deployed their regional e-commerce development strategies to improve the core competitiveness of the regional economy. The rapid development of e-commerce provides a favorable development environment and construction environment for the spatial agglomeration of e-commerce service industry.

## 1. Introduction

While users are using such huge multimedia data more and more, more and more people are using cloud computing technology. It is necessary to effectively manage big data and consider the transmission efficiency of multimedia data of different qualities. A variable allocation algorithm is required for this. This study proposes a method to design a MapReduce scheme applying the FP-growth algorithm, which is a data mining method based on the IaaS (infrastructure as a service) stage of the Hadoop platform, including CPU, network, and storage. The method is then used to allocate resources using this scheme [1]. This study is devoted to applying evolutionary algorithms, gradient methods, and artificial neural networks to the problem of mechanical structure recognition. A dedicated intelligent computing technology (ICT) for global optimization is proposed. ICT is based on a two-phase strategy. The first stage adopts an evolutionary algorithm as a global optimization method. The second stage adopts a special local method combining gradient method and artificial neural network. The proposed technique has many advantages. The key issue of the proposed method is the application of artificial neural networks to compute sensitivity analysis [2]. This study proposes to use the quality prediction method to develop a cloud computing-based intelligent manufacturing scheduling system. A CBIMS continuously builds a variety of different production line layout modes. We use a cloud database for data decentralization and storage, and the scheduling engine contains a sequence scoring system for products, an optimized layout system, and a monitoring system for all available resources [3]. Big data fusion intelligence is the core issue of data science and engineering. This study will first analyze the connotation of big data fusion from the perspective of complex systems. The new research perspective of deep learning technology and the new technology trend of granular processing in data fusion are analyzed, and finally, the architecture of particle computing and processing used to build an intelligent big data integration model for complex system intelligence research is discussed. The research of this subject is a meaningful research and development method in system management and control [4]. According to previous studies, robot walking can only be achieved in prespecified spaces and prespecified actions. In this study, a walking system for a bipedal robot uses fuzzy systems and neural networks to overcome these limitations. The system enables bipedal walking in a variety of environments and more complex obstacles. To do this, a walking robot should recognize its surroundings and determine its movements. In the proposed system, the robot uses neural networks to dynamically generate the walking path of each of its joints as it encounters new obstacles, such as stairs, and maintains walking stability thanks to the control system. The walking stability is maintained by controlling the closed-loop fuzzy control system of the lumbar joint [5]. This article was prepared with financial support from the UK Government's Department for International Development, funding a B2B e-commerce research project in developing countries. The authors draw on comments from Robin Mansell, John Humphrey, and Hubert Schmitz in previous publications in which they collaborated on this research project. Any errors or omissions are the sole responsibility of the authors [6]. We recommend designing an intelligent agent to improve the accessibility of e-commerce applications and websites for the visually impaired. An important feature of this design is the use of information presentation techniques, especially conceptual structures that accurately capture and represent the navigational semantics of each document. It allows users to express high-level navigation destinations using design techniques to achieve these goals. In practice, complex parts of HTML documents are traversed by proxy servers on behalf of visually impaired users [5]. As an emerging network technology, cloud computing provides new methods and means for the construction of e-commerce service system. The author discusses the operation mechanism of the service platform from four aspects: the distributed storage of resources, the coordination of service subjects, and the multiparty interaction between services and security, aiming to promote the rapid development of e-commerce in the cloud computing environment [7]. This study firstly extends log4j and then applies the log file distribution function of log4j to the e-commerce service system. In this way, all log information can be avoided centrally interspersed in a single log file, and log information of different concerns can be effectively dispersed, which is convenient for monitoring and analyzing the running status of the e-commerce service system [8]. Whereas traditional marketing is product-centric, e-commerce marketplaces focus exclusively on customers. The challenge of e-commerce is to really capture the interest of the Internet user and tailor the answer to his requirements that helps the business to target the right customer with the right product or service. To address these issues, the system analyzes the property marketing of online businesses to connect advertisements to target customer groups. Through an agent-based architecture and obfuscation techniques, the system provides simple support for e-commerce market intermediaries [9]. First, a multinomial logit (MNL) model was constructed to reveal the influence of individual attributes, family attributes, and safety hazards on residents' travel satisfaction and to clarify the influencing factors. Then, with significant factors as independent variables, a tourism satisfaction evaluation model based on support vector machine is constructed. The results show that the following factors have a significant impact on residents' travel satisfaction: age, work, education level, number of cars, income, living area, and hidden safety hazards of people, vehicles, roads, and environment [10]. This article conducts a comprehensive and effective survey and data collection on the current situation of geriatric nursing with questionnaires and establishes an evaluation index system that influences the satisfaction of geriatric nursing services with the SERVQUAL model. Based on this, this article analyzes one-dimensional data into two-dimensional data, uses extensive computer vision research, and then uses the educated online model as an effective analysis tool to provide possible predictive outcomes to improve the health care of proposed retirees [11]. Even if neural language models encode these constraints, we design an extensible test suite to address different aspects of utterance and dialogue coherence. Unlike most previous coherence assessment studies, we address language-specific devices beyond sentence order perturbations, allowing for a more fine-grained analysis of what constitutes coherence and what neural models trained on language modeling goals actually encode. This paradigm is equally applicable to assessing the quality of language that contributes to the concept of coherence [12]. The job responsibilities of teachers have changed significantly in recent years, and now more than ever, there is an urgent need for high-quality teachers to achieve the goals of ESD, especially in developing countries. This timely study examined professional and nonprofessional teachers' assessment competencies and their satisfaction [13]. Job satisfaction is one of the most important variables in student standards. We compare, but are not limited to, a number of employee-related variables, including performance, organizational commitment, and core concepts. The results provide documentation of the structural impact and identify two-thirds. The unique effect was found to be the strongest predictor of job satisfaction, despite the use of the satisfaction measure. Further developments are needed to structure the impact, knowledge, and components of these factors and evaluations of job satisfaction predictions [14].

## 2. Research on e-Commerce Services

### 2.1. Deep Docking between e-Commerce Services and Individual Consumers

e-commerce relies on online system platforms to provide users with services of different types and natures. Whether it is purchasing physical products, recharging games in virtual space, or even making lists for fans on specialized service websites, they can all be regarded as the category of e-commerce services. In the era of big data, people in the industry need to expand their management concepts, should not focus on traditional commodities, logistics, and other services, and should summarize all transaction behaviors based on the Internet platform into the e-commerce service system. In the future, enterprises should deeply infiltrate e-commerce into individual consumers, emphasizing individualized services for consumers. Every ordinary consumer is the service object of e-commerce enterprises. Organizations must provide accurate and proactive customer service through scientific analysis of big data. Organizations must also innovate and improve service models in daily consumption and self-satisfaction, such as when consumers buy clothes. They only enjoy the personalized service of premium members; that is, online or offline designers can provide consumers with unique clothing designs. It cannot only enrich the service content but also bring users the ultimate enjoyment and service, so that they can feel the respect and attention from the enterprise. The groups of e-commerce services are shown in Figure 1. The scope of sub-business is very wide and generally can be divided into business-to-business, or business-to-consumer, or two. There is also a consumer-to-consumer model that is growing in stride. As the number of Internet users in China grows, the method of using the Internet to purchase and pay with a debit card is becoming increasingly popular. Market share is also growing rapidly. e-commerce sites are slowly evolving. The most common security mechanisms for e-commerce are SSL (secure socket layer) and SET (secure electronic transaction protocol).

### 2.2. Innovation Strategy of the e-Commerce Service Model

Today, the Internet provides global connectivity. Through the network, customers can bypass distance restrictions and provide consulting and consumption services to global merchants at any time. Despite the growing share of the e-commerce market, the influx of anonymous users has created many problems for the company. With the development of data technology, marketers can accurately identify anonymous shoppers and recommend products that satisfy customers' purchasing power by examining their attention and enthusiasm for purchasing. This not only saves consumer consultation time but also helps merchants avoid the cost of moving unnecessary merchandise. Based on this, providing these services is not enough—e-commerce companies need to improve service specifications and find market gaps from data analysis to service development.

As the online shopping model becomes more and more popular, e-commerce models such as Taobao, Pinduoduo, and Tmall Suning Tesco have shown positive growth. People have a wider choice of shopping routes, and the logistic requirements for these online shopping businesses are also greater. E-commerce businesses not only need to serve customers and recommend products but also need to enhance transportation and logistics. For example, consumers may want to buy their favorite fruit online, but the delivery time is too long and they miss the coldest moment, which naturally makes customers happy. Therefore, enterprises need to evaluate the nature of products purchased by consumers; data technology is used to select the most suitable transportation method to effectively improve logistic efficiency.

Due to the unstable market, e-commerce companies should not copy others' words along the way, and if they see an advantage over other companies, they do not copy them. You will only look ridiculous and never go the way of a market economy. Electronics companies not only focus on this fact in business operations but also make similar mistakes in the field of services. In the era of big data, e-commerce companies can use real-time market analysis to predict future market trends and fine-tune their service models. The e-commerce innovation strategy is shown in Figure 2.

### 2.3. Suggestions for Improving e-Commerce Services

#### 2.3.1. Building a Multilingual Service Platform

Intensification and integration are the focus of cross-border e-commerce service innovation. Cross-border transfers include multilingual communication and customs documentation to complete logistics and distribution; multiple currency changes and multilingual payment instructions are required. A multilingual service platform is established to solve language translation problems.

#### 2.3.2. Providing Full Logistic Services

Cross-border logistic services can improve cross-border e-commerce, making it easier for local consumers to search for information in other countries and buy high-quality, affordable products. Logistic services are provided throughout the process, greatly enhancing cross-border e-commerce opportunities. For example, overseas warehousing and logistic providers bear development costs; speed will combine various transportation methods to meet the needs of different suppliers, including security and after-sales service. The delivery and delivery time of all logistic service products are shortened, and customers with a one-stop solution are provided. It includes product tracking service. Cargo visibility service is a local and international logistic information platform that connects importing companies to provide real-time cargo information. The service aims to accurately understand market demand, help cross-border e-commerce companies to accurately locate goods, and distribute popular science vehicles to increase capacity.

#### 2.3.3. Strengthening Omni-Channel Management

Massive mobile Internet applications have created multichannel channels in the network, expanding the scope of no application boundaries, integrating online and offline, and taking multichannel channels as the development goal. Overseas “tentacles” (such as opening foreign experience stores and opening foreign warehouses through display business) are created to shorten the distance with customers; experience services combined with online product information are provided; customer trust, discounts, and promotions are built; and it is inspiring. Consumption provides value-added services for enterprises. The proposed model of e-commerce service is shown in Figure 3.

## 3. Intelligent Computing Algorithm

### 3.1. Federated Average Algorithm

In traditional machine learning methods, feature extraction needs to capture unique features based on images and unique detection purposes, such as HOG features that emphasize the outline of objects and Haar features that focus on light and dark contrast. After the features are described, they are sent to the machine learning algorithm for classification, such as SVM and AdaBoost, and then determine the classification of objects. The image detection and recognition tasks are completed by performing the sliding frame operation on the image or substituting the above process into the preprocessed ROI frame.

Centralized learning algorithm, distributed learning across devices, learns local model updates and occasionally interacts with a central server to coordinate global learning objectives. Unlike traditional machine learning methods, blended learning requires training models to be centralized on a computer or data center so that each client device can use a local training dataset to update the model. Federated learning is defined as solving the minimization of the objective loss function according to equation (1), where *K* is the total number of client devices and *n*_*k*_ is the number of samples in the dataset on the client device *k*. The combinatorial learning algorithm uses the shared dataset as *n*=∑_*k*_*n*_*k*_ and *p*_*k*_=*n*_*k*_/*n*. It is expressed as the proportion of the total set of algorithm training data for each device *k*.

The data of horizontal federated learning are divided horizontally, and the data schemas of the participants are consistent and have the same characteristics. This is the most mature direction of federated learning at present. The federated learning first proposed and implemented by Google can be regarded as horizontal federated learning, except that the participants are its APP clients.

(1) $$\begin{array}{c} \min\;f\;\left(\omega \right)=\frac{1}{n}\sum_{k=1}^{k}n_{k}F_{k}\left(\omega \right)=\sum_{k=1}^{k}p_{k}\left(\omega \right). \end{array}$$

The local prediction loss function trained by the model parameters for each client device *k* is *F*_*k*_(*ω*), as shown in equation (2). By computing multiple local optima, it is aggregated to achieve global learning loss minimization.

Centralized learning algorithm, distributed learning across devices, learns local model updates and occasionally interacts with a central server to coordinate global learning objectives. Unlike traditional machine learning methods, federated learning requires training models to be centralized in a data center on a machine or computer, allowing each client device to use a local training dataset for model updates. Federated learning is defined to solve the objective loss function minimization.

(2) $$\begin{array}{c} F_{k}\left(\omega \right)=\frac{1}{n_{k}}i\in n_{k}f\left(x_{k;}\omega \right). \end{array}$$

This will improve common patterns in connected learning systems. To solve the objective equation (1), FedAvg first randomly selects *k* units from a subset of system units at each computation iteration and then uses a combined FedSGD optimization method to globally implement each selected unit, computing the sum of the global state and local data.

(3) $$\begin{array}{c} g_{k}=\Delta F_{k}\left(\omega_{k}\right),\\ \forall k,\omega_{t+1}^{k}⟵\omega_{t}-\eta g_{k}. \end{array}$$

In each round of the update round, the server collects training data from all devices participating in that training round of the pattern and calculates the weighted average system update pattern according to equation (4), where *η* represents the training learning rate.

(4) $$\begin{array}{c} \omega_{t+1}⟵\omega_{t}\eta \sum_{k=1}^{k}1. \end{array}$$

The number of elements in the FedAvg algorithm plays a crucial role in the speed of convergence and the accuracy of predictions. Some people suggest adding the stack size to some value to approximate disk. When installing a large compressed package, each device can speed up the calculation of the same amount of data, improve the convergence speed of the system, reduce the number of iterations, and keep the training of the system at a high enough level of accuracy.

### 3.2. Balanced Optimization Algorithm

In the equilibrium optimization algorithm, two points *P*_1_ and *P*_2_ are used within a hypersphere of radius of 1 for local development and global exploration, respectively. The search radius *δ*_1_ based on point *P*_1_ will become smaller and smaller, which has the meaning of shrinking inward, corresponding to the yin, while the search radius *δ*_2_ based on the point *P*_2_ will become larger and larger. It has a sense of outward expansion, which is consistent with any Yang pair. In an intelligent optimization algorithm, local development and global exploration are both complementary and competitive, corresponding to yin-yang mutual root and yin-yang opposition, respectively. In the calculation process, the local search and global search based on points *P*_1_ and *P*_2_ are continuously strengthened, which corresponds to both yin and yang. If point *P*_2_ is better than point *P*_1_, then these two points are exchanged, and the sympathetic algorithm corresponding to yin and yang is repeated based on points *P*_1_ and *P*_1_. The optimization search of *P*_2_ is expected to achieve a balance between local development and global search, corresponding to the balance of yin and yang. In the specific implementation, the yin-yang balance optimization algorithm mainly includes two stages: the solution update based on the archive set and the solution update based on the hypersphere. The main contents of these two stages are given below. The search radius *δ*_1_ and *δ*_2_ are updated, and the calculation method is as follows:

(5) $$\begin{array}{c} \delta_{1}=\delta_{1}-\left(\frac{\delta_{1}}{\alpha }\right),\\ \delta_{2}=\delta_{2}+\left(\frac{\delta_{2}}{\alpha }\right), \end{array}$$

where *α* represents the scaling factor. In this stage, *P*_1_ is the center, *δ*_1_ is the radius, *P*_2_ is the center, and *δ*_2_ is the radius to perform local search and global search in the hypersphere. According to the algorithm design, these two searches use the same solution update equation. For the convenience of expression, let *P* and *δ* denote the search center and radius. Before updating the solution, firstly 2D identical points *P* are generated, denoted by *NP*_1_, *NP*_2_, ⋯*NP*_2*D*_, respectively, and then the update operation on these 2D points is performed. In the algorithm, one component or all components of a point can be updated. A component update equation for a point is as follows:

(6) $$\begin{array}{c} NP=P^{j}+\delta \times \frac{r}{\sqrt{2}},\\ NP=P^{j}+\delta \times \frac{r}{\sqrt{2}},k=D+1,D+2,2D. \end{array}$$

Among them, *NP* represents the *NP* component of point *j*; *P*^*j*^ represents the *P* component of point *r*; and *r* represents the random number between 0 and 1. When updating all components of the point, 2D × *D* is also used. Binary matrix B requires each binary string of the matrix to be unique, and the updated equation for all components of points is as follows:

(7) $$\begin{array}{c} NP_{K}=P^{j}+\delta \times r,B_{k}^{j}=1,\\ NP=P^{j}-\delta \times r,B_{k}^{j}=0, \end{array}$$

where *B*_*k*_^*j*^ represents the matrix element at row *k* and column *j*. In the algorithm, one of the above two update methods is selected with a probability of 50%. It has the characteristics of strong fine-tuning ability and applies wavelet to the learning of these elite solutions. Let *X* be an elite solution in the file set, and the new solution after learning through the wavelet elite solution is *X*^*∗*^. The specific method is as follows:

(8) $$\begin{array}{c} X^{*}=\gamma X+r\left(L+U\right). \end{array}$$

Among them, *γ* is the wavelet function value; *r* is a random number between 0 and 1; and *U* and *L* are the upper and lower bounds of the variable *X*. Because the Morlet wavelet has excellent time-frequency characteristics and dynamic characteristics, it is a typical representative of the dynamic change space of wavelet function, this study will use the Morlet wavelet in the calculation of equation (8), and its calculation method is as follows:

(9) $$\begin{array}{c} \gamma =\frac{1}{\sqrt{a}}\exp\left(1{\left(\frac{\Phi }{2}\right)}^{2}\right)\cos\left(5\left(\frac{\Phi }{2}\right)\right),\\ a=\exp\left(-\ln\;g\times {\left(1-\frac{t}{T}\right)}^{\xi }\right)+\ln\;g. \end{array}$$

Among them, *g* represents the upper bound of a; *t* represents the current number of iterations of the algorithm; *T* represents the maximum number of iterations; ξ represents the shape parameter. In the algorithm, the elite solution retained in the archives is compared with the new solution learned by adopting the wavelet elite solution, and the best two solutions to *P*_1_ and *P*_2_ are assigned_,_ respectively. In addition, if these elite solutions are local optimal solutions, the learning of these solutions can also jump out of the local extreme points to avoid premature convergence of the algorithm.

*g* represents the upper bound of a; *t* represents the current number of iterations of the algorithm; *T* represents the maximum number of iterations; ξ represents the shape parameter. In the algorithm, the elite solution retained in the archives with the new solution learned by adopting the wavelet elite solution is compared, and the best two solutions to *P*_1_ and *P*_2,_ respectively, are assigned.

### 3.3. Lightweight MobileNet-SSD Model Construction

To adapt to the computing power limitation of embedded devices, this study constructs the MobileNet-SSD network, adopts the lightweight MobileNet feature extraction network, combines it with the SSD detection network, and replaces the backbone network VGG-16 in the SSD with MobileNet, which greatly reduces the memory usage. Then, patches of different scales and aspect ratios are placed a priori on the feature maps of different scales, and the predicted boundary patches are based on the previous patch. The size of the previous image depends on the scale and aspect ratio. The rules for scaling the previous frame in different target maps are as follows:

(10) $$\begin{array}{c} S_{k}=S_{\min}+\frac{S\max-S_{\min}}{M-1}\left(k-1\right),\;k\in \left[1,m\right]. \end{array}$$

In the formula, the *K*th feature map of *S*_*k*_ shows the relationship between the size of the previous frame and the feature map; *S*_min_ and *S*_max_ represent the maximum and minimum values, respectively; *m* represents the number of map features. From equation (10), it can be seen that as the map feature size decreases, the scale of the previous field increases linearly. This article predefines the aspect ratio of the box according to the prior configuration rules of the SSD box:

(11) $$\begin{array}{c} a_{r}\in \left\{1,2,3,\frac{1}{2},\frac{1}{3}\right\}. \end{array}$$

In the formula, *a*_*r*_ is the aspect ratio of the prior frame. According to the aspect ratio and the scale of the a priori frame, the width and height of the prior frame are calculated, and the calculation formula is as follows:

(12) $$\begin{array}{c} w_{k}^{a}=s_{k}\sqrt{a_{r}},\\ h_{k}^{2}=\frac{s_{k}}{\sqrt{a_{r}}}, \end{array}$$

where *w*_*k*_^*a*^ and *h*_*k*_^2^ are the width and height of the prior frame, respectively. The loss of the whole process is divided into two parts, the weighted sum of the position loss and the confidence loss, that is, the loss function. The input sample *x* is defined, and then, the loss function is defined as follows:

(13) $$\begin{array}{c} L\left(x,c,l,g\right)=\frac{1}{n}\left(L_{\text{conf}}\left(x,c\right)\right)+\alpha L_{\text{conf}}\left(x,c,l,g\right),\\ Pe\left(Q\left(K+1\right)\right)=S_{i}Q\left(k\right)=s_{j}. \end{array}$$

In the formula, *c* is the trust value of the trust class; *l* is the predicted value of the associated box position corresponding to the previous box; *g* is the position parameter of the actual object; and *N* is the number of positive samples in the previous field. Finally, non-maximum suppression (NMS) is used to reduce the number of negative samples. Since multiple multiscale feature maps will generate a large number of prior frames, which contain a large number of redundant and overlapping samples, resulting in redundant computation, NMS can be used to perform iterations the traversal-elimination process filters the a priori boxes, which can effectively improve the network performance.

## 4. Prediction and Evaluation of e-Commerce Services

### 4.1. e-Commerce Service Evaluation Index of Intelligent Computing

We summarized the questions in the questionnaire and came up with 10 secondary indicators. These include the secondary indicators of the customer service index system, the popularity and satisfaction of customer service attitudes, the speed, safety, attitude, price, and other indicators of secondary logistic services. By analyzing the indicator system, we are satisfied with the logistics of Shentong. Some categories are listed in Tables 1 and 2.

Among them, in the establishment of the merchant satisfaction evaluation index system, the first-level index is the merchant's satisfaction, and the second-level indicators are the merchant's after-sales service, the merchant's reputation, and the attitude of the merchant's customer service; in the establishment of the logistic satisfaction evaluation index system, we found that the satisfaction of logistics is the first-level indicator, and the second-level indicators are the speed of logistics, the safety of logistics, the service attitude of logistics, and the price of logistics.

When establishing an index system to measure seller satisfaction, the survey questions are summarized into first-level indicators, and the second-level indicators are salesperson service, salesperson popularity, and salesperson attitude. Dealer customer service: when establishing the logistic satisfaction index system, we found that logistic satisfaction is the first-level indicator, and the second-level indicators are logistic speed, logistic safety, service logistic ratio, and logistic price. The data collected can be used to assess customer satisfaction with services, popularity, customer service, logistic speed, security, and service and trade logistic prices. “Very satisfied” represents 5 points, “satisfied” represents 4 points, “generally satisfied” represents 3 points, “dissatisfied” represents 2 points, and “very dissatisfied” represents 1 point; the 5-year total score of each indicator is calculated on the basis of annual satisfaction. By calculation, we get Figure 4.

Through the analysis of Figure 4, we find that the membership degree also increases with the increase in the year, which indicates that the evaluation of the e-commerce service is getting better and better each year. Through the increase in the year, we also find that the weighted average satisfaction has been increasing the rate of increase and membership increase in 2019–2020 is the fastest, indicating the highest e-commerce satisfaction in this year.

### 4.2. Prediction of e-Commerce Service Satisfaction Based on Intelligent Computing

It can be seen from the following figure that there is not much difference between the predicted value and the actual value, indicating that the e-commerce service satisfaction prediction is effective. In 2018, the actual comprehensive score of service satisfaction was 2.8, the prediction of polynomial fitting was 2.9, and the prediction of Gaussian curve fitting was 2.98; in 2019, the actual comprehensive score of service satisfaction was 3.2, the prediction of polynomial fitting was 3.26, and the prediction of Gaussian curve fitting was 3.2. The forecast is 3.3; the actual comprehensive score of service satisfaction in 2020 is 3.9, the polynomial fitting forecast is 3.81, and the Gaussian curve fitting forecast is 3.86; in 2021, the actual comprehensive score of service satisfaction is 4.5, and the polynomial fitting forecast is 4.56. Gaussian curve fit predicts 4.44, as shown in Figure 5.

The model can help e-commerce service platforms to quickly judge the indicators that affect satisfaction. Through the gradual regression results of the satisfaction prediction model, the improvement of indicators such as after-sales service, customer service attitude, and logistic speed, safety, service attitude, and logistic price can be obtained. It can improve service satisfaction. The fitting result of stepwise regression analysis is *R*^2^ = 0.9996, indicating that the model has a high degree of fit, as shown in Table 3.

### 4.3. Comparison of Service Accuracy under Intelligent Computing

In this article, we use the intelligent computing method to calculate the e-commerce service satisfaction evaluation, which improves the accuracy of the effect evaluation. In order to obtain the evaluation of e-commerce service satisfaction under intelligent computing, the intelligent computing method is compared with other computing methods in accuracy. We conducted a comparison test, and the comparison results are shown in Figure 6:

According to the experimental data of the figure, we can know that the evaluation accuracy of the algorithm after intelligent calculation is the highest among the three methods. When the number of times reaches 40, the evaluation accuracy of the intelligent algorithm can reach about 0.9, and when the number of times reaches 30, in the three methods the accuracy of the algorithm is the closest to around 0.5.

### 4.4. Performance Test

The performance advantages of the intelligent algorithm technology model proposed in the article are tested. The test will test the models of the three algorithms proposed in the article. The smart algorithm is an ambiguous statistical algorithm and the pseudo-algorithm model runs on a test suite and an integrated test suite, respectively. The test suite is used to evaluate the general capabilities of the final model. A set of hybrid tests is used to tune the model's hyperparameters, and initially, the model's capabilities are evaluated. The results of the tests are recorded to verify the validity of the three sample ratings. A curve according to the test results is drawn.

According to the data in the table and graph, we can conclude that after running on the test set, the model accuracy rate of the fuzzy statistical algorithm can reach 89.12%, the accuracy rate can reach 89.56%, the accuracy rate of the intelligent algorithm can reach 92.46%, and the accuracy rate can reach 92.46%. It reaches 93.27%, which is the highest index value among the three experimental models. The accuracy of the artificial model is 75.14%, which is the lowest among the three systems, and the fuzzy statistical model is in the middle state. According to the curves of the three algorithms, we can also see that the curve values of the intelligent computing and fuzzy statistical algorithm models are very stable, and the experimental results also show that the performance of the intelligent computing algorithm is the best, as shown in Table 4 and Figure 7.

According to the data in Table 5 and Figure 8, after running the hybrid test package, the performance of the three models decreases somewhat, but the performance of the smart computer model is still high. In three models, the accuracy rate of the fuzzy statistical algorithm is 87.25%, and the accuracy rate of the intelligent computer algorithm is 90.12%. According to the performance of the three algorithms, it can be seen that the intelligent computer algorithm is very stable and always at 0.95, whether it is a test set or a mixed test set. The experimental results also show that the model validation accuracy of the intelligent computing algorithm is very high.

## 5. Conclusion

Through the comparison of algorithms and experiments, we can conclude that the current e-commerce services are facing severe postgraduate entrance examinations, and more and more e-commerce platforms are facing the risk of bankruptcy. In the face of these risks, government departments should introduce corresponding measures, such as introducing corresponding policies to reduce the taxation of merchants; the government should relax the corresponding import and export of goods. Our experiments in the fourth part can be concluded that, after running on the test set, the model accuracy rate of the fuzzy statistical algorithm can reach 89.12%, the accuracy rate can reach 89.56%, the accuracy rate of the intelligent algorithm can reach 92.46%, and the accuracy rate can reach 93.27%, which is one of the highest index values in the experimental model.

## Figures and Tables

**Figure 1:** e-commerce service groups.

**Figure 2:** e-commerce innovation strategy.

**Figure 3:** e-commerce service suggestion.

**Figure 4:** Weighted average satisfaction.

**Figure 5:** Fitting comparison between actual and predicted values of e-commerce service satisfaction.

**Figure 6:** Comparison of evaluation accuracy.

**Figure 7:** Curve of the test set.

**Figure 8:** Performance on the mixed test set.

**Table 1:** Establishment of the evaluation index system of merchant satisfaction.

First-level indicator	Secondary indicators	Symbol
Merchant satisfaction	After-sales service	H1
	Reputation	H2
	Customer service attitude	H3

**Table 2:** Establishment of the evaluation index system of logistic satisfaction.

First-level indicator	Secondary indicators	Symbol
Logistic satisfaction	Logistic speed	T1
	Safety	T2
	Service attitude	T3
	Logistic price	T4

**Table 3:** Stepwise regression analysis results of the service satisfaction prediction model.

Secondary indicators	Analysis results		
	Correlation coefficient	*P* value	Salience
After-sales service	0.273	0.03	Significant
Reputation	0.028	0.105	Not obvious
Customer service	0.309	0.0169	Not obvious
Logistic speed	0.021	0.0298	Not obvious
Safety	0.0294	0.0076	Not obvious
Service attitude	0.243	0.0243	Not obvious
Logistic price	0.225	0.0345	Not obvious
Fitting results	Intercept = 1.154	*R* ^2^ = 0.9996	

**Table 4:** Performance of each model on the test set.

Model	Accuracy (%)	Accuracy (%)	Score (%)
Fuzzy statistical algorithm model	89.12	89.56	90.48
Intelligent algorithm model	92.46	93.27	93.45
Artificial algorithm model	85.45	85.43	86.18

**Table 5:** Performance of each algorithm on the mixed test set.

Model	Accuracy (%)	Accuracy (%)	Score (%)
Fuzzy statistical algorithm model	87.88	87.12	88.96
Intelligent algorithm model	90.12	90.24	90.29
Artificial algorithm model	82.14	82.47	82.64

## Data Availability

The experimental data used to support the findings of this study are available from the corresponding author upon request.

## References

[1] Kaplinsky R. G. (2000). Unequalisation: What can Be learned from value chain analysis. *Journal of Development Studies*.

[2] Seongu L., Heejun (2006). Intelligent Walking of a Biped Robot Using Soft-Computing Method. *Information and Control Symposium*.

[3] Deng W., Rong C., Yang X. (2010). An intelligent fault diagnosis method based on soft computing and expert system. *International Journal of Engineering Intelligent Systems for Electrical Engineering & Communications*.

[4] Choi J., Choi C., Yim K., Kim J., Kim P (2013). Intelligent reconfigurable method of cloud computing resources for multimedia data delivery. *Informatica*.

[5] Pontelli E., Son T. C. (2004). Designing intelligent agents to support universal accessibility of E-commerce services [J]. *Electronic Commerce Research and Applications*.

[6] Pushpalatha M., Kathiravan A. V.

[7] Xu J., Hsu V. N., Niu B. (2018). The impacts of markets and tax on a multinational firm’s procurement strategy in China. *Production and Operations Management*.

[8] Liu W. Z., Tao Q. Y., He Q., Yu L. J (2014). Application of Log4j in E-commerce services. *Applied Mechanics and Materials*.

[9] Loia V., Senatore S., Sessa M. I. (2008). Customized advertising in E-commerce services provision. *éè·è*.

[10] Xu Z., Shao C., Wang S., Dong C (2020). Analysis and prediction model of resident travel satisfaction. *Sustainability*.

[11] Gao J., Song J., Han L. (2021). Research on analysis and prediction of elderly medical satisfaction based on convolutional neural network. *Journal of Physics: Conference Series*.

[12] Kook H., Lee (2010). Prediction and evaluation of indoors noise level of exhibition room in museum by road traffic noise. *Journal of Korean Society of Environmental Engineers*.

[13] Chen Y., Liu Y., Zhang M. (2017). Predicting User Satisfaction in SERPs with Mouse Movement Information. *IEEE Transactions on Knowledge & Data Engineering*.

[14] Monika A. (1997). Wisdom and life satisfaction in old age. *J Gerontol B Psychol, Soc*.

